# Efficacy of Bushen Yiqi Huayu Decoction on Ovarian Reserve and Inflammatory Factors in Patients after Hysterectomy plus Salpingectomy

**DOI:** 10.1155/2022/5866685

**Published:** 2022-03-02

**Authors:** Jinchun Zhang, Li Zhang, Lei Cao

**Affiliations:** ^1^Department of Obstetrics, Qingdao Municipal Hospital (Group), Qingdao, Shandong, China; ^2^Department of Obstetrics and Gynecology, Beijing Hospital of Integrated Traditional Chinese and Western Medicine, Beijing, China; ^3^Maternal and Child Health Hospital, Shanghai, China

## Abstract

**Objective:**

To assess the efficacy of Bushen Yiqi Huayu Decoction on ovarian reserve and inflammatory factors in patients after hysterectomy plus salpingectomy.

**Methods:**

Between January 2020 and December 2020, sixty patients with benign uterine lesions scheduled for a hysterectomy plus salpingectomy in the obstetrics and gynecology department of our hospital were recruited and assigned at a ratio of 1 : 1 via the random number table method to receive conventional therapy (control group) or conventional therapy plus Bushen Yiqi Huayu Decoction (study group) for 2 months. The traditional Chinese medicine (TCM) symptom scores, TCM efficacy, various postoperative recovery time indexes, inflammatory factor levels, and hormone levels were compared between the two groups of patients.

**Results:**

The study group had lower TCM symptom scores and milder inflammatory responses compared to the control group after treatment (*P* < 0.05). The Bushen Yiqi Huayu Decoction plus conventional therapy achieved an efficacy of 96.67% versus the efficacy of 76.67% by conventional therapy alone (*P* < 0.05). In contrast to the control group, a shorter postoperative recovery duration of patients was recorded in the study group (*P* < 0.05). The study group showed significantly better improvement in hormone levels than the control group after treatment (*P* < 0.05).

**Conclusion:**

Bushen Yiqi Huayu Decoction can significantly mitigate the inflammatory response of patients after hysterectomy plus salpingectomy, improve the hormone level and the ovarian reserve of patients, and promote rapid recovery, so it is worthy of clinical promotion.

## 1. Introduction

Hysterectomy is currently a common treatment for benign uterine pathologies including fibroids and endometrial polyps [1]. Recent studies have found that concomitant removal of the ovaries during a hysterectomy may reduce the risk of postoperative ovarian cancer in patients with benign uterine disease to some extent and may not exacerbate the ovarian decline in the immediate postoperative period [2,3]. However, the concurrent hysterectomy with salpingectomy may compromise ovarian reserve and thus aggravate perimenopausal symptoms in patients [4]. It has also been reported that postoperative inflammatory response is one of the essential factors affecting the rapid recovery of patients after hysterectomy plus salpingectomy [5]. According to TCM, postoperative patients may develop negative emotions due to their loss of the uterus and ovaries, resulting in liver qi discomfort and qi blockage. In addition, intraoperative blood loss can lead to the intermingling of blood deficiency and blood stasis and postoperative deficiency of the kidney essence biochemistry, resulting in the deficiency of kidney [6]. TCM treatment should be performed based on the principles of tonifying the kidney, benefiting qi, and resolving stasis in a dialectical manner [7]. Accordingly, Bushen Yiqi Huayu Decoction was used for patients scheduled for a hysterectomy plus salpingectomy to explore its efficacy. The results are as follows.

## 2. Materials and Methods

### 2.1. General Information

Between January 2020 and December 2020, sixty patients with benign uterine lesions scheduled for a hysterectomy plus salpingectomy in the obstetrics and gynecology department of our hospital were recruited and assigned via the random number table method to a control group (*n* = 30) or a study group (*n* = 30). Inclusion criteria were as follows: (1) patients aged 35–55 years without fertility plans; (2) patients with normal preoperative menstrual cycle without perimenopausal symptoms; (3) patients with no tubal lesions confirmed by preoperative vaginal ultrasound; and (4) patients those who received hysterectomy plus salpingectomy successfully. Exclusion criteria were as follows [8,9]: (1) patients with preoperative menopause; (2) patients with a history of previous obstetrical and gynecological surgery; (3) patients receiving sex hormone therapy 3 months before surgery; (4) patients with other serious medical diseases or gynecological inflammatory diseases such as pelvic inflammatory disease or vaginitis or serious organ tissue disorders, psychiatric diseases, or immune system diseases. The study was approved by the ethics committee of the hospital and was performed under supervision, and all patients provided written informed consent.

### 2.2. Methods

Patients in the control group were given conventional postoperative interventions. Patients were given antibiotics within 3 days after surgery and were instructed to eat easily digestible and light foods. Tub bathing was prohibited for 2 weeks after surgery, and sexual intercourse was not allowed for 1 month after surgery, with attention to hygiene and early out-of-bed activities [10].

On the basis of the treatment of the control group, the study group additionally adopted the Bushen Yiqi Huayu Decoction [6,11,12]. The recipe includes 20 g Poria; 15 g each of Rhizoma Atractylodis Macrocephalae, Radix Codonopsis Pilosulae, Radix Rehmanniae Praeparata, Endothelium Corneum Gigeriae Galli, and Radix Angelicae Sinensis; 12 g Pinellia Tuber; 10 g each of Radix Paeoniae Alba, Rhizoma Ligustici Chuanxiong, and peach seed; and 6 g each of safflower, Radix Bupleuri, tangerine peel, and prepared liquorice root, with 1 dose/day. Each dose was divided in half and orally administered in the morning and evening, respectively. The treatment spanned 2 months.

### 2.3. Outcome Measures

(1) TCM symptom score: symptoms include abnormal menstrual flow, lower abdominal pain, abnormal menstrual periods, abnormal leucorrhea, weakness of Qi, yellowish complexion, and fever. The TCM symptom score was evaluated as follows: 6 points: severe symptoms, 4 points: moderate symptoms, 2 points: mild symptoms, and 0 points: the absence of adverse symptoms [13]. (2) TCM efficacy: the effectiveness of TCM was evaluated as per the degree of reduction in the evaluation results of TCM symptom score. The TCM efficacy was evaluated as follows: markedly effective: a reduction in the index of more than 70%; effective: a reduction in the index of between 30% and 70%; ineffective: a reduction in the index of less than 30% or aggravation. (3) Postoperative recovery time indicators: recovery time of bowel sounds, exhaustion time, defecation time, time of pain disappearance, and time of menstruation recovery. (4) Inflammatory factors: tumor necrosis factor-*α* (TNF-*α*) and interleukin-6 (IL-6). Before and after treatment, 5 ml of peripheral venous blood was collected from the eligible patients after the menstrual period, and a double-antibody sandwich enzyme-linked immunosorbent assay was used to determine the levels of TNF-*α* and IL-6. (5) Hormone level: hormone indices include luteinizing hormone (LH), follicle-stimulating hormone (FSH), estradiol (E2), and progesterone. Before and after treatment, 5 ml of fasting venous blood was collected from the patients on the 2nd–3rd day of menstruation, and the above indexes were determined by using an enzyme-linked immunoassay.

### 2.4. Statistical Analyses

The data were analyzed using SPSS 26.0 statistical software. The measurement data were expressed as mean ± standard deviation ($\bar{x}\pm \text{s}$), and the *t*-test was used for comparison between two groups. The count data were expressed as (*n* (%)), and the *χ*2 test was used for comparison between groups. The difference was considered statistically significant at *P* < 0.05.

## 3. Results

### 3.1. Comparison of Baseline Data

There was no statistically significant difference in age, operation time, intraoperative bleeding, menstrual cycle, BMI, type of disease, type of operation, parity, and education levels between the two groups (*P* > 0.05) (Table 1).

### 3.2. Comparison of TCM Symptom Scores

The two groups presented no great disparity in TCM symptom scores before treatment (*P* > 0.05). After treatment, the study group obtained significantly lower TCM symptom scores compared to the control group (*P* < 0.05) (Table 2).

### 3.3. Comparison of TCM Efficacy

The TCM efficacy of the study group was 96.67%, which was remarkably higher than that of the control group (76.67%) (*P* < 0.05) (Table 3).

### 3.4. Comparison of Postoperative Recovery Time

A shorter postoperative recovery time of various indicators was recorded in the study group in contrast to the control group (*P* < 0.05) (Table 4).

### 3.5. Comparison of Inflammatory Factor Levels

Before treatment, no significant statistical difference in inflammatory response indexes between the groups was found (*P* > 0.05). After treatment, the inflammatory response indexes of the study group were significantly lower than those of the control group (*P* < 0.05) (Table 5).

### 3.6. Comparison of Hormone Level

The two groups did not differ in terms of hormone level before treatment (*P* > 0.05). After treatment, the study group showed significant improvement in the hormone level indicators as compared to the control group (*P* < 0.05) (Table 6).

## 4. Discussion

Previous research has found [14] that the uterus, ovaries, and fallopian tubes are more liable to experience pathological changes, which are considered to be related to female hormone disorders. Surgical treatment is the mainstay for the radical cure of such lesions. However, notwithstanding the active use of minimally invasive surgery in the treatment of such diseases, surgical damage to patients is still unavoidable [15]. The ovary is an important female reproductive organ, and its decreased reserve function significantly compromises female fertility. Laparoscopic hysterectomy plus salpingectomy may cause abnormal ovarian blood supply and superovulation due to the absence of the fallopian tubes in a short period of time, compromising ovarian reserve and decreasing ovarian responsiveness [16]. In TCM, kidney deficiency and blood stasis are considered to be the underlying pathogenesis of postoperative ovarian reserve decline in hysterectomy plus salpingectomy patients. It has been reported that cleansing the heart, nourishing the kidney, and strengthening the spleen can effectively alleviate perimenopausal symptoms and signs and delay the process of ovarian function decline in posthysterectomy patients [17].

The Bushen Yiqi Huayu Decoction is a homemade formula made in our hospital with reference to relevant literature and clinical experience. In this formula, Radix Rehmanniae Praeparata nourishes Yin and tonifies the kidney, safflower invigorates the blood and dispels stasis, Radix Codonopsis tonifies the Middle Jiao, strengthens the spleen, and nourishes the blood, and they constitute the monarch drugs. Radix Angelicae Sinensi tonifies the blood, Rhizoma Atractylodis Macrocephalae and White Paeony Root tonify the blood and relieve pain, and Rhizoma Ligustici Chuanxiong invigorates the blood and promotes menstruation, which were the ministerial medicines. Peach kernel and safflower invigorate blood circulation and eliminate blood stasis, Radix Bupleuri detoxifies the liver and relieves depression, Poria strengthens the spleen and nourishes the heart, tangerine peel regulates the qi and strengthens the spleen, and Radix Glycyrrhizae Preparata harmonizes all the herbs. The combination of the above medicines works to tonify the kidneys, benefit the qi, and remove blood stasis. The results of this study showed that the TCM symptom score, TCM efficacy, postoperative recovery time indexes, inflammatory response indexes, and hormone levels were substantially improved after the application of Bushen Yiqi Huayu Decoction combined with conventional postoperative interventions in patients undergoing hysterectomy and salpingectomy. According to TCM [14], the main pathogenesis of patients undergoing hysterectomy and salpingectomy is Qi deficiency and blood stasis, with the main pathological features as deficiency of positive Qi and unexhausted phlegm and stasis. Such pathology undermines the recovery of the patient's gastrointestinal function after surgery and produces adverse symptoms such as pain, abnormal menstruation, and emotional disorders, affects hormone levels and inflammation levels, and increases the risk of postoperative infections [18,19]. Therefore, the present study applied Bushen Yiqi Huayu Decoction in the adjuvant treatment of patients after hysterectomy plus salpingectomy to investigate its efficacy to further determine its application value.

The total efficacy of the study group was 96.67%, which was significantly higher than that of the control group (76.67%), and the TCM symptom scores showed that the TCM symptom scores of patients in both groups were significantly reduced after treatment, and the TCM symptom scores of the study group were significantly lower than those of the control group, suggesting that the addition of Bushen Yiqi Huayu Decoction on top of conventional treatment can help alleviate the TCM symptoms and signs of patients with high treatment efficiency, which is worthy of clinical application. In addition, the significantly shorter postoperative recovery time in patients given Bushen Yiqi Huayu Decoction suggests that the decoction contributes to the rapid recovery of patients. Research has shown that hysterectomy plus salpingectomy may impair ovarian reserve and compromise ovarian responsiveness in patients in the short term [16]. Another study revealed a strong correlation between conventional basal endocrine hormone levels and ovarian reserve [20]. In the present study, LH, FSH, E2, and P levels were found to be significantly lower in both groups after treatment, and the study group had significantly lower levels of the above indicators than the control group after treatment, suggesting that the addition of Bushen Yiqi Huayu Decoction can improve the ovarian reserve of patients after surgery by improving hormone levels [21]. Serum TNF-*α* and IL-6 levels were significantly reduced in both groups after treatment, with more significant reductions in the study group, suggesting a therapeutic effect of Bushen Yiqi Huayu Decoction on inflammation after hysterectomy plus salpingectomy. The detailed mechanism requires further investigation.

In conclusion, Bushen Yiqi Huayu Decoction can significantly mitigate the inflammatory response of patients after hysterectomy plus salpingectomy, improve the hormone level and the ovarian reserve of patients, and promote rapid recovery, so it is worthy of clinical promotion. The limitations of this study lie in the small sample size and short follow-up period, which prevented the determination of changes in ovarian function in patients 6 months or even 1 year postoperatively and may result in some bias. Future studies with expanded sample size and longer follow-up are proposed to further clarify the application of Bushen Yiqi Huayu Decoction in the postoperative treatment of patients undergoing hysterectomy plus salpingectomy.

## Figures and Tables

**Table 1:** Comparison of baseline data.

Items	Study group (*n* = 30)	Control group (*n* = 30)	*t*/*χ*^*2*^	*P*
Age (years)	45.52 ± 6.81	45.64 ± 6.78	0.068	0.946
Operation time (min)	85.14 ± 9.93	84.38 ± 9.87	0.297	0.767
Intraoperative bleed (ml)	39.81 ± 15.15	40.24 ± 15.21	0.110	0.913
Menstrual period (d)	29.43 ± 4.24	29.36 ± 2.25	0.080	0.937
BMI (kg/m^2^)	25.38 ± 4.23	25.34 ± 4.26	0.036	0.971

Type of disease				
Uterine fibroids	12	12	1.089	0.780
Endometrial polyps	8	6		
Functional uterine hemorrhage	5	8		
Adenomyosis	5	4		

Type of surgery				
Hysterectomy with bilateral salpingectomy	10	12	0.287	0.592
Hysterectomy with unilateral salpingectomy	20	18		

Parity				
0	8	7	0.315	0.854
1	18	20		
≥2	4	3		

Education level				
Elementary school and below	5	4	0.302	0.860
Middle school	19	21		
Junior college and above	6	5		

**Table 2:** Comparison of TCM symptom scores ($\bar{x}\pm \text{s}$).

Groups	Case (*n*)	Before treatment	After treatment
Control group	30	25.24 ± 4.36	12.52 ± 5.84
Study group	30	25.15 ± 3.92	8.76 ± 6.50
*t*	—	0.084	2.356
*P*	—	0.933	0.021

**Table 3:** Comparison of TCM efficacy (*n*(%)).

Groups	Case (*n*)	Markedly effective	Effective	Ineffective	Total effective rate
Control group	30	10 (33.33)	13 (43.33)	7 (23.33)	23 (76.67)
Study group	30	11 (36.67)	18 (60.00)	1 (3.33)	29 (96.67)
*χ* ^2^	—	—	—	—	5.192
*P*	—	—	—	—	0.022

**Table 4:** Comparison of postoperative recovery time ($\bar{x}\pm \text{s}$).

Groups	Case (*n*)	Recovery time of bowel sounds (h)	Exhaustion time (h)	Defecation time (d)	Time of pain disappearance (d)	Time of menstruation recovery (d)
Control group	30	25.27 ± 5.66	72.47 ± 6.44	3.16 ± 1.32	5.27 ± 2.44	38.27 ± 9.77
Study group	30	18.96 ± 6.84	50.47 ± 7.23	1.43 ± 0.63	2.78 ± 1.96	26.46 ± 9.97
t	—	3.892	12.445	6.478	4.357	4.634
*P*	—	≤0.001	≤0.001	≤0.001	≤0.001	≤0.001

**Table 5:** Comparison of inflammatory response indexes ($\bar{x}\pm \text{s}$).

Groups	Case (*n*)	TNF-*α* (ng/L)		IL-6 (ng/L)	
		Before treatment	After treatment	Before treatment	After treatment
Control group	30	85.54 ± 5.63	38.98 ± 3.57	35.39 ± 4.45	16.95 ± 2.64
Study group	30	85.28 ± 5.65	31.36 ± 3.34	34.90 ± 5.23	10.42 ± 2.53
*t*	—	0.178	8.537	0.390	9.781
*P*	—	0.858	≤0.001	0.697	≤0.001

**Table 6:** Comparison of hormone level ($\bar{x}\pm \text{s}$).

Groups	Case (*n*)	LH (mIU/ml)		FSH (mIU/ml)		E2 (pg/ml)		Progesterone (ng/ml)	
		Before treatment	After treatment	Before treatment	After treatment	Before treatment	After treatment	Before treatment	After treatment
Control group	30	63.29 ± 8.75	46.18 ± 7.63	18.16 ± 0.82	12.54 ± 0.69	126.58 ± 0.85	75.20 ± 0.83	13.38 ± 1.37	7.38 ± 1.68
Study group	30	62.86 ± 6.52	41.63 ± 7.28	18.24 ± 0.59	10.46 ± 0.93	126.66 ± 0.94	64.93 ± 0.58	13.26 ± 1.19	5.92 ± 1.53
*t*	—	0.215	2.363	0.433	9.838	0.345	55.552	0.362	3.519
*P*	—	0.829	0.021	0.666	≤0.001	0.730	≤0.001	0.718	≤0.001

## Data Availability

No data were used to support this study.
